# Teachers’ emotional exhaustion before and during the COVID-19 pandemic: Neither emotional exertion nor vacation feeling

**DOI:** 10.3389/fpsyg.2022.887494

**Published:** 2022-08-08

**Authors:** Victoria Bleck, Frank Lipowsky

**Affiliations:** Department of Empirical Educational Research, Institute of Educational Science, Faculty of Human Sciences, University of Kassel, Kassel, Germany

**Keywords:** Coronavirus disease, emotional exhaustion, in-service-teachers, latent-change, longitudinal study, teacher stress

## Abstract

**Purpose:**

In this paper, we use latent change models to examine the changes in in-service teachers’ emotional exhaustion before and during the COVID-19 pandemic. As a result of the pandemic, teachers are confronted with challenging tasks, which can lead to stress and burnout. Resultingly, teachers’ stress experiences have been examined in different studies. However, often the *change* in those experiences remains unclear. Against this background, we investigate longitudinally how the emotional exhaustion of a cohort of German teachers changes. In addition, we examine whether gender, age, teaching degree studied, or the amount of time spent in distance learning affected the change during the pandemic.

**Methods:**

We surveyed German veteran teachers (*N* = 382) about their emotional exhaustion at three measurement points. The first two surveys were before the COVID-19 pandemic (*t*_1_: winter 2016/2017; *t*_2_: spring: 2019), and the third measurement point was after the first lockdown Germany in summer 2020 (*t*_3_). To answer the research questions, we used neighbor-change models.

**Results:**

Emotional exhaustion increased between the first two measurement points (*t*_1_, *t*_2_) but decreased in the following period (*t*_2_, *t*_3_). The changes in the two periods did not differ significantly from each other. Neither gender, age, nor the teaching profession studied influenced the change in emotional exhaustion. The hours spent in distance learning were also not a significant predictor.

**Conclusion:**

In summary, the COVID-19 pandemic does not appear to be associated with higher emotional exhaustion across the veteran teachers. However, there are some teachers whose emotional exhaustion rises to high levels. Those teachers deserve special attention.

## Introduction

Since the beginning of 2020, the COVID-19 pandemic has had multiple impacts on all aspects of daily life. The educational sector has also been extensively affected by the restrictions associated with the pandemic. All around the world, schools were closed – also in Germany. The associated challenges represented an additional stressor for teachers (Rabaglietti et al., 2021; Weißenfels et al., 2022). Within a short time, they had to convert their lessons to digital formats (König et al., 2020; Lorenz et al., 2020). Following the lockdown, many teachers practiced a mixture consisting of face-to-face instruction at school and homeschooling (Klapproth et al., 2020). At the same time, many felt insecure about digital teaching (Hansen et al., 2020).

Various studies have already captured the perspective of children and parents on the COVID-19 pandemic (e.g., Adams et al., 2021; Bussières et al., 2021; Simm et al., 2021). However, despite teachers’ central role, investigations have less frequently focused on their experiences. This paper addresses the exhaustion of teachers in Germany. In contrast to previous studies, however, the change in emotional exhaustion is examined longitudinally. The first two measurement points were in winter 2016/2017 and spring 2019 – before the COVID-19 pandemic. A third measurement point was during the pandemic in summer 2020.

The study had three purposes. *First*, it investigated whether emotional exhaustion increased or decreased over time. *Second*, it examined whether emotional exhaustion changed differently during the COVID-19 pandemic, in comparison to before the pandemic. *Third*, we tested the influence of gender, age, and teaching degree on the change in emotional exhaustion.

### Emotional exhaustion

Emotional exhaustion represents the central dimension of burnout and describes a feeling of being emotionally overextended and depleted of one’s resources. It manifests as a lack of energy (Maslach et al., 2001) and develops individually differently – depending on person and environment (Lazarus and Folkman, 1984). Thus, depending on their own internal and external resources, different individuals may evaluate the same situation quite differently. While one person views a situation as a challenge that can be mastered, another person might perceive an imbalance of demands and resources and consequently experience the same situation as a threat (e.g., Antonovsky, 1987; Bakker and Demerouti, 2008). Although evaluation is individual, new and unpredictable situations with low subjective controllability are thought to intensify the experience of stress (Lazarus and Folkman, 1984). Consequences are the experience of emotional exhaustion and, in the long term, burnout (Maslach et al., 2001).

To date, some studies provide information on how teachers’ stress and burnout change throughout their professional lives. Generally, occupational stress seems to be a largely stable construct as far as the mean value is concerned (Hultell, 2011). In other words, emotional exhaustion scarcely increases or decreases across all participants in a sample. Even over 16 years, teachers’ experienced job strain does not vary significantly on average (Bleck et al., 2019). However, changes in emotional exhaustion are evident for beginning teachers (Hultell et al., 2013; Dicke et al., 2016) and during teacher induction (in German *Referendariat*; Dicke et al., 2015; Voss and Kunter, 2020). Although the effect sizes are small, emotional exhaustion increases at the beginning of teacher induction time and decreases with growing teaching experience throughout the traineeship (Voss and Kunter, 2020). A frequently mentioned explanation for the increase at the beginning is the wide range of new tasks and that teachers are responsible for their lessons and student learning for the first time (e.g., Dicke et al., 2015).

### Emotional exhaustion during the COVID-19 pandemic

The situation during the COVID-19 pandemic is associated with unpredictability and low controllability for everyone, especially for teachers. In this respect, the experience of emotional exhaustion could increase, comparable to the career entry experiences. In interviews, teachers in England were asked about their feeling about the COVID-19 pandemic and described uncertainty about the future as a central theme (Kim and Asbury, 2020; Kim et al., 2022). Argentine teachers stated in a survey that uncertainty about the consequences of the COVID-19 pandemic was the greatest stressor for them (Vargas Rubilar and Oros, 2021). Teachers in Germany have also reported feelings of uncertainty (Hansen et al., 2020). At the same time, demands and resources for coping with everyday professional life are changing (Hilger et al., 2021). Even if occupational demands and resources were in balance before the COVID-19 pandemic, resources might no longer be sufficient to cope with the lockdown requirements and the associated homeschooling (Weißenfels et al., 2022). Against this background, it is also plausible to assume that teachers’ emotional exhaustion increases during the pandemic.

Whether in the United Kingdom, Italy, Vietnam, or Germany, the perceived workload of teachers in many places around the world has increased due to COVID-19 (e.g., Giovannella et al., 2020; Hansen et al., 2020; See et al., 2020; Vu et al., 2020). The heavier workload arises, among other things, from the additional organizational and communication requirements, and from initial familiarization issues with digital media (forsa, 2020). This perceived workload could also be associated with increased emotional exhaustion. Results from Canada suggest that teachers are having higher levels of stress and emotional exhaustion during the COVID-19 pandemic (Sokal et al., 2020b). The values were above the theoretical mean. Teachers from the United States, Spain, and Finland also reported high levels of stress, burnout, and negative emotions (Ozamiz-Etxebarria et al., 2021; Pöysä et al., 2021; Chang et al., 2022). However, a study of German teachers found a decrease in workload and fatigue after the first lockdown (Hilger et al., 2021). Filipino teachers’ mental health appears to have been little affected by the COVID-19 pandemic (Rabacal et al., 2020). While one-third of teachers have low levels of perceived stress, only one in 10 Filipino teachers surveyed in August 2020 reported high levels of stress (Oducado et al., 2021). A study in Israel found that teachers reported experiencing more burnout than before the COVID-19 pandemic (Gutentag and Asterhan, 2022). Teachers in the United Kingdom also showed high levels of well-being, although around half of the survey respondents experienced online teaching as stressful (See et al., 2020).

Prior studies in German-speaking countries have also focused on stress and occupational strain among teachers during the COVID-19 pandemic. Results of the school barometer (Huber and Helm, 2020) indicate that around 40% of school staff felt very stressed 2 weeks after the beginning of the first lockdown in March 2020. A representative survey of 310 teachers conducted in April 2020 shows that most teachers were coping well with the new situation (Eickelmann and Drossel, 2020). However, teachers’ perceived stress during the pandemic varied greatly: On the one hand, around one-third reported feeling less stressed than usual. These were mainly teachers who did *not* provide digital services during school closures. On the other hand, one-third of the respondents felt more stress than usual – regardless of their gender or age. One in six teachers felt overwhelmed by the new situation during the pandemic (Eickelmann and Drossel, 2020).

Using a sample of teachers from the German federal state Thuringia (*N* = 1.263), Dreer and Kracke (2021) show that their participants’ job satisfaction during the lockdown in April 2020 was high and that the teachers felt moderately stressed. Hansen et al. (2020) also summarize that the teachers they surveyed show a high occupational satisfaction – despite the pandemic. Nevertheless, at the same time, the authors point out that one in four teachers show symptoms of burnout. In the survey conducted by Lorenz et al. (2020) in April and May 2020, the teachers also described both positive and negative emotions. The teachers’ perceived occupational stress was at a medium level. However, a higher level was reported by the female teachers in the sample and by teachers who did not feel sufficiently supported by the school management. In another cross-sectional study with teachers of different school types in Germany, the respondents reported a medium or high level of stress: They sometimes or often felt nervous or strained during the 4 weeks prior to taking part in the survey (Klapproth et al., 2020). The perceived stress was greater among female teachers than among male teachers and also greater among high-track secondary school teachers compared to those in other types of schools. In addition, the study showed a correlation between the experienced stress and the time spent daily on distance learning.

The mentioned studies indicate that, during the COVID-19 pandemic, German teachers are experiencing challenges associated with increased emotional exhaustion (see also Eickelmann and Drossel, 2020; Klapproth et al., 2020). However, the studies did not take into account the emotional exhaustion pre-pandemic, making the reported values difficult to interpret. Furthermore, most studies only focused on the *state* of stress and exhaustion but did not survey any *change*. There are a few exceptions to this restriction. In a qualitative study, 24 teachers were interviewed at various times during the COVID-19 pandemic (Kim et al., 2022). The authors conclude that mental health and well-being appear to decline during the period. Lindner et al. (2021) found a decrease in job satisfaction among Austrian teachers until the first lockdown. During this period, female teachers’ job satisfaction declined more than the satisfaction of male teachers. However, job satisfaction before the pandemic was only examined retrospectively during the COVID-19 pandemic.

In the following, we report the results of quantitative studies that analyzed changes in well-being and stress before and during the COVID-19 pandemic. A study with Chilean teachers showed a significant decrease in life satisfaction from pre-pandemic to summer 2020 (Lizana et al., 2021). Pellerone (2021) questioned teachers from Italy about their feelings of burnout. Her findings indicate that teachers rated their personal performance as a dimension of burnout significantly lower during the pandemic compared to an earlier survey. The general level of burnout was significantly higher, although there were no significant changes in emotional exhaustion and depersonalization. A recent study from Germany by Weißenfels et al. (2022) examined the changes in burnout and self-efficacy based on data from 92 teachers. The first survey was conducted in fall 2019, with the second survey starting in May 2020. Using latent change models, the authors show that, while lack of accomplishment and depersonalization increased significantly, emotional exhaustion did not. Sokal et al. (2020a) surveyed Canadian teachers at two measurement points *during* the pandemic – in April 2020 and June 2020. Over the investigation period during the pandemic, both teachers’ emotional exhaustion and depersonalization increased.

Unfortunately, the studies that have investigated change in emotional exhaustion did not have the data to compare the change before and during the pandemic. Thus, this longitudinal survey depicting and comparing long-term changes – before and during the COVID-19 pandemic – can provide data about essential to interpreting findings related to teachers’ emotional exhaustion.

### Research questions

Up to now, only a few studies describe the change in teachers’ emotional exhaustion during the COVID-19 pandemic. Exceptions are the described studies conducted by Sokal et al. (2020a), Lizana et al. (2021), Pellerone (2021), and Weißenfels et al. (2022). Despite their longitudinal design, it is unclear how the change in emotional exhaustion during the pandemic differs from the change before the pandemic. The first research question of the paper arises from this lack of corresponding studies:

*Research question 1:* Has teachers’ emotional exhaustion changed differently in times of the COVID-19 pandemic in comparison to before the pandemic?

The challenges for teachers associated with the pandemic are often emphasized. These challenges may be linked to a higher workload and increased emotional exhaustion. However, previous studies also show that the experience of teachers varies greatly: While some teachers report increased stress, a similarly high proportion of teachers report experiencing less stress than before the pandemic (Eickelmann and Drossel, 2020). Due to the inconsistent findings, we do not formulate a hypothesis about the change in emotional exhaustion. Instead, the aim is to test whether the emotional exhaustion that changed between spring 2019 and summer 2020 (during the COVID-19 pandemic) was similar to the change between the two measurement points before the COVID-19 pandemic.

In a second step, to learn more about the change in emotional exhaustion during the COVID-19 pandemic, we examine the regression of stress change on gender, age, and teaching profession studied. In addition, we investigate if the time spent in distance learning predicts the change of emotional exhaustion during the pandemic.

*Research question 2*: Do gender, age, the teaching profession studied, and the amount of time spent in distance learning predict the interindividual change in emotional exhaustion?

We developed two hypotheses related to this research question. Some research findings on *gender* suggest that female teachers experience higher occupational stress and emotional exhaustion than male teachers (Klapproth et al., 2020; Lorenz et al., 2020; Lindner et al., 2021; Oducado et al., 2021; Ozamiz-Etxebarria et al., 2021). In contrast, Eickelmann and Drossel (2020) report that the experience of occupational stress varies among teachers regardless of their gender. The relation between *age* and the experience of stress has been less frequently studied. Previous research suggests no association between the two characteristics (Eickelmann and Drossel, 2020; Oducado et al., 2021). A correlation between age and stress was found only in the retrospective study by Jakubowski and Sitko-Dominik (2021). In the study conducted by Weißenfels et al. (2022), the change in emotional exhaustion was independent of teachers’ gender and work experience.

While Lorenz et al. (2020) found that the *type of school* also does not affect the perceived occupational stress, the results from Klapproth et al. (2020) suggest that teachers at high-track secondary schools are more stressed than teachers at other types of schools. However, the present sample does not include participants who have studied teaching for high-track secondary schools. Therefore, a hypothesis is only formulated for gender while investigating the influence of age and teaching degree in an exploratory manner.

*Hypothesis a*: Emotional exhaustion increases significantly more among female teachers than among male teachers.

The change to digital teaching is associated with numerous challenges for many teachers and became a particular stressor during the pandemic. In this respect, we assume that digital teaching has a higher potential for emotional exhaustion than other teaching practices more similar to conventional lessons. On the other hand, if teachers do not conduct digital lessons during school closures, the workload should also be reduced. Thus, it is not surprising that Eickelmann and Drossel (2020) found that teachers who did not provide digital resources felt less stressed. Furthermore, the extent to which they teach digitally seemed to influence the emotional experience. Teachers who spent more hours a day on distance learning reported higher occupational stress (Klapproth et al., 2020). In this respect, we formulate the following assumption for the interrelation between the amount of time spent in distance learning and the change in emotional exhaustion:

*Hypothesis b*: The more hours teachers spent on distance learning per week, the higher the increase in emotional exhaustion during the COVID-19 pandemic.

## Materials and methods

The data are part of the longitudinal project *professional paths* (in German *Wege im Beruf*; Lipowsky, 2003; Bleck et al., 2019). The project focuses on former students of Universities of Education in the German federal state Baden-Württemberg who completed their teacher education program between 1995 and 1997. Besides teachers, the sample also comprises graduates working outside the teaching profession. From 1999 to now, they were assessed 12 times on their professional situation and their professional experiences. Thus, the project has been running for over 20 years. Over time, the content focus has evolved and changed. As a result, not all constructs have been measured at all time points. However, some constructs like occupational stress were included in all surveys.

This paper focuses on the teachers in the sample and uses the data from three survey dates. We examined the change in emotional exhaustion starting from winter 2016/2017 (*t*_1_) through spring 2019 (*t*_2_). These time points are thus *before* the start of the COVID-19 pandemic. The third assessment point was in summer 2020 (*t*_3_) and therefore was conducted *during* the pandemic. Data was collected using an online questionnaire.

### Sample

The total sample consists of 977 graduates who participated in the first two surveys in 1999 and 2001. The following analyses include all participants from whom data are available for at least one of the three measurement points (*N* = 505). Participants working outside the teaching profession at one of the three measurement points were excluded from the analyses (*N* = 123). Accordingly, 382 teachers remain in the sample. At the last measurement point in summer 2020, the participants were on average 51 years old (*M* = 50.53, *SD* = 2.92) and had worked for about 20 years in the teaching profession (*M* = 20.04, *SD* = 3.24). Accordingly, this is a group of veteran teachers.

They taught mainly in grades 5–9 (52.1%) or 1–4 (46.9%). They have studied primary and low-track secondary school teaching (*Grund- & Hauptschullehramt*, 61.8%) or middle-track secondary school teaching (*Realschullehramt*, 38.2%). The average teaching load was around 21 h (*M* = 20.53, *SD* = 6.06) with a real working time of around 31 h per week (*M* = 30.86, *SD* = 12.91).

The final sample participants (*N* = 382) do not differ from the rest of the original sample (non-participants: *N* = 595) either in the teaching profession studied (χ^2^(1) = 1.52, *p* = 0.218), in gender (χ^2^(1) = 1.21, *p* = 0.271) or in year of birth (*t*(934.81) = −1.87, *p* = 0.062). There are also no differences between participants and non-participants in occupational stress at the first measurement point in the project (2001; *t*(707) = −0.86, *p* = 0.392) or at the last time of measurement before 2016 (*t*_1_), which was in 2012 (*t*(390) = −0.28, *p* = 0.783).

As participants without complete data are also considered in the longitudinal analysis, data are missing at particular measurement points. The percentage of missing values is 20.2% at *t*_1_ in winter 2016/2017 and 15.7% at *t*_2_ in spring 2019. At *t*_3_, the survey during the COVID-19 pandemic, 23.8% of the data are missing. Since there are also missing values for some variables, the proportion of missing values is up to 28.0% per measurement. To handle the missing data, we performed multiple imputation using the package mice (van Buuren and Groothuis-Oudshoorn, 2011) in R 3.6.2. We generated 20 imputed data sets that are included for the analyses.

### Measures

We used a German adaption (Enzmann and Kleiber, 1989) of the Maslach Burnout Inventory (Maslach et al., 1996) to assess emotional exhaustion at three measurement points. Participants were asked: “We are interested in how you experience your employment. Please rate the extent to which the following statements apply to you.” The four items (e.g., “I often feel exhausted at work”) have a Likert format ranging from 1 *does not apply at all* to 7 *applies completely*.

First, we tested the measurement invariance of the instrument at three measurement points. Strict measurement invariance is considered a prerequisite for testing differences in means (van de Schoot et al., 2012). Table 1 shows the fit indices of the models with different degrees of measurement invariance. In the models, correlations of the residuals of the same items at different measurement times were allowed (correlated uniqueness; Marsh and Hau, 1996). The model of *configural invariance* (without restrictions) shows a good model fit. The model fit remains stable even when equating the factor loadings in the *metric invariance* model (ΔCFI < 0.01, ΔRMSEA < 0.015; Cheung and Rensvold, 2002). Equating the intercepts in the *scalar invariance* model leads to a decrease in model fit, but the differences remain below the cut-offs (ΔCFI < 0.01, ΔRMSEA < 0.015; Cheung and Rensvold, 2002). Therefore, the instrument has the necessary level of strict measurement invariance over time.

**Table 1:** Series of CFA models investigating measurement invariance of emotional exhaustion.

	χ^2^/*df*	*p*(χ^2^)	CFI	TLI	RMSEA	AIC
Configural invariance	2.07	<0.001	0.973	0.954	0.053	15,463.03
Metric invariance	1.96	<0.001	0.972	0.959	0.050	15,554.35
Scalar invariance	2.04	<0.001	0.965	0.955	0.052	15,473.01

We had already asked about gender (1 *female*, 2 *male*), birth year, and the teaching profession studied (1 *primary and low-track secondary school teaching*, 2 *middle-track secondary school teaching*) at an earlier measurement point in the project. How many hours per week the teachers spent on distance learning was determined at *t*_3_ with the question: “On average, how many lessons per week have you conducted distance learning since mid-March?” On average, the teachers held around 10 lessons per week digitally (*M* = 9.97, *SD* = 7.14).

### Analyses

To investigate our research questions, we specified latent change models in Mplus 7. Latent change models capture changes dynamically and directly in structural equation models (McArdle, 2009). Latent difference variables were modeled, representing interindividual differences in the change in emotional exhaustion on a latent level. The mean and variance of the latent difference score can be tested for significance, and predictor variables can be included in the models (Steyer et al., 1997; McArdle, 2009). The model fit was assessed using the fit indices commonly used for structural equation models. Thus, to avoid misinterpretation, we used different fit indices – χ^2^ as well as CFI, TLI, and RMSEA – to estimate the model fit. χ^2^ depends on sample size and leads to significant values in larger samples (Chen, 2007). Therefore, we consider χ^2^ concerning the degrees of freedom. Both CFI and TLI have proven useful for assessing the model fit and should be ≥0.90 for an acceptable fit. Values ≥0.95 suggest a good fit to the data (Hu and Bentler, 1999; Brown, 2006). For RMSEA, values ≤0.08 suggest an acceptable fit, and values <0.05 indicate a good fit (Brown, 2006).

To answer *research question 1*, we specified a neighbor-change model based on the strict measurement invariance model. The model contains the differences between the first and second measurement time point (*t*_1_, *t*_2_) and between the second and third measurement time point (*t*_2_, *t*_3_). To test whether the changes differ significantly, the intercepts of the latent difference variables were set equal in the next step. A Chi-square test was used to check whether the restricted model fits significantly worse than the model without restrictions. To answer *research question 2*, we included additional covariates in the model to predict the baseline value and the two latent difference scores.

## Results

### Changes in emotional exhaustion

With *research question 1*, we investigate how emotional exhaustion has changed before and during the COVID-19 pandemic. Are the changes similar or significantly different? To answer the question, we specify a neighbor-change model (χ^2^/*df* = 1.91, *p*(χ^2^) < 0.001; CFI = 0.97, TLI = 0.96, RMSEA = 0.05, AIC = 15,468). The latent baseline score of emotional exhaustion is below the theoretical mean (*M* = 2.83; Table 2). Consequently, at the first measurement point (*t*_1_, winter 2016/2017), the teachers felt emotionally exhausted to a relatively low degree. The latent difference between this first and the second measurement point in spring 2019 (*t*_2_–*t*_1_) is positive and significant (*M* = 0.12, *SE* = 0.06, *p* = 0.041). This result indicates that emotional exhaustion increased significantly in the sample between the two measurement points *before* the COVID-19 pandemic. Given that the variance of the latent difference score is also significant (*σ* = 0.68, *SE* = 0.11, *p* < 0.001), emotional exhaustion varies substantially between the teachers.

**Table 2:** Means and variances of the latent variables.

	Means (*M*)	Variances (*σ*)
Latent baseline score (*t*_1_)	2.83 (*SE* = 0.06), *p* < 0.001	1.91 (*SE* = 0.16), *p* < 0.001
Latent difference (*t*_2_–*t*_1_)	0.12 (*SE* = 0.06), *p* = 0.041	0.68 (*SE* = 0.11), *p* < 0.001
Latent difference (*t*_3_–*t*_2_)	−0.05 (*SE* = 0.06), *p* = 0.367	0.54 (*SE* = 0.09), *p* < 0.001

The latent difference between the second and third measurement time points (*t*_3_–*t*_2_) reveals the change in emotional exhaustion from spring 2019 to summer 2020. The intercept of the latent difference is negative (*M* = −0.05, *SE* = 0.06). Across all teachers in the sample, emotional exhaustion decreased slightly over about 1 year, including the beginning of the COVID-19 pandemic. However, the difference score and thus the change in emotional exhaustion is not significant (*p* = 0.367). Once again, the variance of the latent difference score indicates individual differences in the change in emotional exhaustion (*σ* = 0.54, *SE* = 0.09, *p* < 0.001).

While emotional exhaustion increased significantly in the period *before* the COVID-19 pandemic (from *t*_1_ to *t*_2_), emotional exhaustion does not change significantly in the following period, including the beginning of the pandemic (from *t*_2_ to *t*_3_). However, if we equate the intercepts of the latent difference scores, the Chi-square difference test yields no significant difference compared to the model with freely estimated parameters (baseline model: χ^2^(59) = 112.79, *p* < 0.001; restricted model: χ^2^(60) = 115.83, *p* < 0.001; Δχ^2^ = 3.04, Δ*df* = 1, *p* = 0.081). Therefore, the change in emotional exhaustion is comparable over both periods.

The change in emotional exhaustion between the first two measurement points (*t*_2_–*t*_1_) is significantly negatively related to the baseline score at t_1_ (*r* = −0.36, *p* < 0.001). Those teachers with high emotional exhaustion at the first measurement point tended to experience a decrease in emotional exhaustion up to the second measurement point. In contrast, the change between the second and third measurement point is not significantly related to the latent baseline score (*r* = −0.15, *p* = 0.066).

### Predictors of emotional exhaustion

In the next step, gender, year of birth, and teaching profession studied were simultaneously included as predictors for the baseline value of emotional exhaustion and the latent differences. The hours teachers spent in distance learning each week are modeled only as a predictor of the change in emotional exhaustion from *t*_2_ to *t*_3_, as it is a feature of the pandemic. Table 3 reports the standardized regression coefficients of the model (χ^2^/*df* = 1.52, *p*(χ^2^) < 0.001; CFI = 0.97, TLI = 0.96, RMSEA = 0.04, AIC = 15,478).

**Table 3:** Prediction of the baseline score and the latent differences in the neighbor-change model.

	Latent baseline score		Latent difference (*t*_2_–*t*_1_)		Latent difference (*t*_3_–*t*_2_)	
	*β* (*SE*)	*p*	*β* (*SE*)	*p*	*β* (*SE*)	*p*
Gender^1^	−0.07 (0.06)	0.296	0.07 (0.07)	0.338	−0.02 (0.09)	0.802
Year of birth	−0.02 (0.06)	0.758	0.00 (0.08)	0.956	−0.05 (0.10)	0.608
Teaching profession studied^2^	−0.06 (0.06)	0.314	0.03 (0.08)	0.731	−0.06 (0.09)	0.468
Distance learning	–		–		0.06 (0.07)	0.382

1 One female, two male.

2 One primary and low-track secondary school teaching, two middle-track secondary school teaching.

The baseline level of emotional exhaustion in winter 2016/2017 was slightly higher among female teachers than among male teachers, but the difference is not significant (*β* = −0.07, *p* = 0.296), nor is the subsequent change in emotional exhaustion predicted by gender (*t*_2_–*t*_1_: *β* = 0.07, *p* = 0.338; *t*_3_–*t*_2_: *β* = −0.02, *p* = 0.802). *Hypothesis a*, that emotional exhaustion increases to a greater extent in female teachers than male teachers during the COVID-19 pandemic, must be rejected.

We also tested the influence of the year of birth and the teaching profession. However, neither of the variables shows a significant influence on the baseline value of emotional exhaustion (see Table 3). Furthermore, the latent differences (*t*_2_–*t*_1_, *t*_3_–*t*_2_) are not explained by either of the two variables. The experience of emotional exhaustion at the first measurement point and the change between the subsequent measurement points are therefore independent of birth year and teaching profession studied.

Finally, we examined the influence of the time teachers spent on distance learning each week on the change in emotional exhaustion between spring 2019 and summer 2020. We assumed that emotional exhaustion increased to a greater extent when teachers spent more hours on distance learning (*hypothesis b*). However, the result suggests that this hypothesis must also be rejected (*β* = 0.06, *p* = 0.382).

## Discussion

The COVID-19 pandemic and its consequences are omnipresent. Besides the economic consequences, the consequences in the field of education are receiving much attention. Homeschooling is not only challenging for students and parents; the teachers’ work has also been affected by the pandemic-related changes in schools. In this respect, educational research is focusing on teachers’ experience of stress and emotional exhaustion during the pandemic. However, there is a lack of longitudinal research on the change in teachers’ emotional exhaustion. In addition to existing studies, in this paper, we compared the change in emotional exhaustion before the COVID-19 pandemic with the change during the pandemic.

### Summary

*Research question 1* focused on the change in emotional exhaustion. From winter 2016/2017 to spring 2019 – throughout around 2 years even before the COVID-19 pandemic – the emotional exhaustion of the teachers surveyed increased significantly. From spring 2019 to summer 2020, which includes the start of the pandemic and the first lockdown, however, emotional exhaustion decreased slightly, albeit not significantly.

The situation of teachers caused by the COVID-19 pandemic is characterized by novelty and unpredictability. Therefore, the situation could increase the experience of stress and emotional exhaustion. In line with these theoretical assumptions, evidence was found in a sample of Canadian teachers that teachers’ emotional exhaustion increased from April to June 2020 (Sokal et al., 2020a). On the other hand, there are also results showing that emotional exhaustion has not necessarily increased due to the COVID-19 pandemic. Pellerone (2021) and also Weißenfels et al. (2022) found no evidence of a significant increase in emotional exhaustion among teachers. This insignificant finding also seems to apply to the present sample. It is plausible that the emotional exhaustion of some teachers increases while the emotional exhaustion of other teachers decreases. As a result, no significant change emerges on average. Some teachers reported noticeably extra loads in earlier studies, while a similarly high proportion reported experiencing less stress (Eickelmann and Drossel, 2020). An indicator for such individual differences in change is the variance of the latent difference in our study, which is significantly different from zero (*σ* = 0.54, *SE* = 0.09, *p* < 0.001).

An open question is how these differences in the changes can be explained (*research question 2*). For this purpose, we included socio-demographic data such as gender, year of birth, and the teaching profession studied in the model. Contrary to expectations, gender had no significant effect on emotional exhaustion at the first measurement point (winter 2016/2017). Similarly, the subsequent change up to the second measurement point and the change between the second and third measurement points were unrelated to gender. Subsequently, we rejected *hypothesis a*. As a result, emotional exhaustion in the study sample – similar to Weißenfels et al. (2022) – is independent of teacher gender. Nonetheless, in the literature, gender differences in stress experience are widely reported (e.g., Purvanova and Muros, 2010; Innstrand et al., 2011; Fernet et al., 2012; Skaalvik and Skaalvik, 2016), even during the COVID-19 pandemic (e.g., Klapproth et al., 2020; Lorenz et al., 2020; Oducado et al., 2021). Neither age nor teaching profession studied are significant predictors of emotional exhaustion or its change.

*Hypothesis b* tested whether emotional exhaustion during the pandemic increases with the number of hours teachers spent on distance learning. For example, Eickelmann and Drossel (2020) showed that the experience of stress is higher among teachers with distance learning. More hours in distance learning are also associated with a higher stress experience (Klapproth et al., 2020). However, the change in emotional exhaustion in the present study cannot be explained by the extent of distance learning. This lack of a relationship between the two factors could be related to the time of the survey in the summer of 2020; teachers no longer only taught distance learning but also taught in the classroom. On the other hand, it is conceivable that a high distance learning level only causes stress under certain conditions. A high level of stress could arise if, at the same time, the amount of face-to-face teaching is high or if the teachers believe their competencies for implementing distance learning are low.

### Limitations

When interpreting the results, special attention should be paid to the date of the third *measurement point* during the COVID-19 pandemic. The data collection took place from the end of July 2020 to late October 2020. Pandemic-related restrictions were lower during this phase than during the spring 2020 lockdown. In addition, the summer holidays were during this period. Previous research suggests positive effects of vacations on well-being and dimensions of burnout. However, these effects fade out within a few days or weeks after the vacation (de Bloom et al., 2009). This *vacation effect* is also evident among teachers (e.g., Kühnel and Sonnentag, 2011; Kellmann and Heidari, 2020; Horan et al., 2021). Interviews with teachers indicate that recovery from vacations is lower for middle-aged and older teachers than for younger ones (Skaalvik and Skaalvik, 2015). Although we surveyed a sample of veteran teachers, it seems conceivable that the emotional exhaustion was even higher a few weeks earlier. However, there was no difference in emotional exhaustion between teachers who participated in the survey during holidays (*M* = 3.17, *SD* = 1.29, *N* = 132) and teachers who participated outside of holidays at the third measurement point (*M* = 3.06, *SD* = 1.45, *N* = 138, *t*(268) = −0.67, *p* = 0.502). Additionally, we could not find a significant correlation between the date of survey participation – measured by the week after the start of the survey – and emotional exhaustion at *t*_3_ (*r* = 0.06, *p* = 0.356).

A positive aspect is that the more extended study periods of one to 2 years make it possible to compare changes before and during the COVID-19 pandemic. Nevertheless, it would also be interesting to compare changes during the pandemic within shorter periods. It is conceivable, for example, that emotional exhaustion increased at the beginning of the lockdown and decreased afterward. However, this cannot be stated based on our data. Further, it should be noted that the time between the first and second measurement point (*t*_1_: winter 2016/2017; *t*_2_: spring 2019) is about 2 years, which is about twice as long as the period between the second and third measurement point (*t*_3_: summer 2020). The primary reason for this is that we conducted the third survey *ad hoc* in order to be able to capture the teachers’ experience during the pandemic.

Moreover, unique features of the *sample* must be taken into account. The sample consists of veteran teachers from three consecutive cohorts. In this respect, the sample is relatively homogeneous regarding age and professional experience and is not representative of all teachers in Germany. Even if the conducted dropout analysis (see section Sample) did not indicate, selection bias might have occurred over the long term of the project.

In particular, the differences between various types of schools cannot be represented. Since the teachers completed their first state examination at German Universities of Education in the federal state Baden-Württemberg, the sample does not include graduates for high-track secondary schools. However, the emotional exhaustion of high-track secondary teachers could differ from primary and lower- and middle-track secondary school teachers. According to the findings from Klapproth et al. (2020) high-track secondary teachers felt more stressed than other teachers during the COVID-19 pandemic.

Finally, it should be noted that we used a general version of the Maslach Burnout Inventory (Maslach et al., 1996) to assess emotional exhaustion. The Educator Survey of the Maslach Burnout Inventory (MBI-ES) specifically measures teacher burnout. Although the Educator Survey is more appropriate for the sample of teachers, we used the general version because all participants – including the graduates working outside the teaching profession – were asked about their emotional exhaustion.

### Implications

For research, the study findings raise two central questions. First, the question arises of how emotional exhaustion will continue as the COVID-19 pandemic progresses. Will it decrease as the situation for teachers normalizes, or will it increase? In the study by Sokal et al. (2020a) with Canadian teachers, both emotional exhaustion and depersonalization of teachers increased from April to June 2020. Jakubowski and Sitko-Dominik (2021) also reported increased mental health problems in a sample of Polish teachers. However, the change between the beginning of the COVID-19 pandemic and the winter of 2020/2021 was not significant. Regardless of general trends regarding an increase or decrease in emotional exhaustion, it is crucial to identify those teachers whose emotional exhaustion increases significantly. The consequence can be impairments in motivation or subjective or objective health (Hakanen et al., 2006). Furthermore, the quality of (digital) teaching and students’ learning can also suffer (Klusmann et al., 2008b, 2016).

Additionally, the question arises as to which characteristics can explain the individual change in emotional exhaustion. In the present study, neither gender, nor age, nor teaching profession studied, nor amount of distance learning significantly predicted the latent differences in emotional exhaustion. In addition to occupational demands, occupational and personal resources are also relevant in experiencing situations (Bakker and Demerouti, 2008; Sokal et al., 2020b). For *occupational demands*, time management, dealing with technology, and working with parents are significant predictors of emotional exhaustion during the pandemic (Sokal et al., 2020b). In lockdown times, *private demands*, such as caring for children in homeschooling and family-work conflicts, could also be highly important (Hilger et al., 2021; Gutentag and Asterhan, 2022; Kim et al., 2022). As a limitation, it should be noted that the same requirements do not necessarily have to be associated with the same experiences (Lazarus and Folkman, 1984).

Many studies have identified *social support* as an essential resource (e.g., Bakker and Demerouti, 2008; Voss and Kunter, 2020). Several studies show that support from school leadership, colleagues, and family and friends, is linked to lower emotional exhaustion (e.g., Klusmann et al., 2008a; Skaalvik and Skaalvik, 2016; Wolgast and Fischer, 2017; Voss and Kunter, 2020). During the pandemic, social support – from school leadership, colleagues, or in the private environment – is also considered highly relevant (Sokal et al., 2020b; Jakubowski and Sitko-Dominik, 2021; Kim et al., 2022). For example, teachers who experience their school leadership as autonomy-supportive report less burnout and emotional exhaustion (Collie, 2021; Chang et al., 2022). Further research should examine which type of social support is helpful for teachers during the COVID-19 pandemic. It is conceivable that, similar to teacher induction time, teachers’ instrumental support is especially beneficial (Voss and Kunter, 2020). Accordingly, the exchange of materials and literature seems to be of greater relevance in how prospective teachers experience emotional exhaustion than is the emotional support of peers. Similarly, during the pandemic, teachers could benefit from an exchange of teaching materials and content on methods and tools within the teaching staff.

Finally, *personal resources* are theoretically also crucial in the experience of emotional exhaustion. In this respect, self-efficacy as a resource is associated with the change in emotional exhaustion (e.g., Dicke et al., 2015). Studies also examine the extent to which teachers’ knowledge can protect them from burnout (Lauermann and König, 2016). It seems reasonable, that under the current circumstances of the COVID-19 pandemic, technical knowledge and its application in the classroom (*TPACK*; Mishra and Koehler, 2006) are important in how emotional exhaustion is experienced. For example, Gutentag and Asterhan (2022) found a negative correlation between online teaching proficiency and burnout. Another study shows that the emotional exhaustion of teachers who have participated in a 14-week training on stress management, emotional intelligence, and the use of digital media develops more favorably compared to that of a control group (Pozo-Rico et al., 2020). Thus, teacher training seems to be a resource to protect against emotional exhaustion. Despite the findings of Pozo-Rico et al. (2020), however, it is unclear whether emotional exhaustion is reduced by stress management, emotional intelligence, digital media, or a combination of all three. In the study by Weißenfels et al. (2022), the change in emotional exhaustion is independent of self-efficacy for using digital media and attitudes toward e-Learning.

This study examined the change in emotional exhaustion before and during the COVID-19 pandemic using latent change models. The results show that emotional exhaustion increased significantly over the 2 years *before* the pandemic. However, emotional exhaustion slightly decreased in the following year, including the beginning of the pandemic and the first lockdown. Consequently, coping with the situation during the COVID-19 pandemic was *not* an emotional exertion for the sample of veteran teachers. However, it should be noted that there are substantial differences between teachers, and some of them do report increased emotional exhaustion. Those teachers deserve special attention to avoid burnout and health problems in the long term.

## Data availability statement

The datasets presented in this article are not readily available because the project is not yet completed. The data will be used for further publications and final theses. Requests to access the datasets should be directed to VB (victoria.bleck@uni-kassel.de).

## Ethics statement

Ethical review and approval was not required for the study on human participants in accordance with the local legislation and institutional requirements. The patients/participants provided their written informed consent to participate in this study.

## Author contributions

FL supervised the project and reviewed the manuscript critically. FL and VB designed and administered the surveys. VB drafted the manuscript and performed the calculations. Both authors contributed to the article and approved the submitted version.

## Funding

The project is financed by own funding.

## Conflict of interest

The authors declare that the research was conducted in the absence of any commercial or financial relationships that could be construed as a potential conflict of interest.

## Publisher’s note

All claims expressed in this article are solely those of the authors and do not necessarily represent those of their affiliated organizations, or those of the publisher, the editors and the reviewers. Any product that may be evaluated in this article, or claim that may be made by its manufacturer, is not guaranteed or endorsed by the publisher.
